RETRACTED

# Src-homology domain 2 containing protein tyrosine phosphatase-1 (SHP-1) directly binds to proto-oncogene tyrosine-protein kinase Src (c-Src) and promotes the transcriptional activation of connexin 43 (Cx43)

**DOI:** 10.1080/21655979.2022.2079252

**Published:** 2022-06-05

**Authors:** YiHao Liu, Meng Dai, PengHui Yang, Li Cao, Li Lu

**Affiliations:** a Department of Cardiovascular Medicine, Children’s Hospital of Chongqing Medical University, Chongqing, China; b Department of Palliative Medicine, Chongqing University Cancer Hospital, Chongqing, China; c Department of Cardiology, the Second Affiliated Hospital of Chongqing Medical University, Chongqing, China; d Department of Critical Care Medicine, University-Town Hospital of Chongqing Medical University, Chongqing, China

**Keywords:** HL-1 cells, Cx43, SHP-1, c-Src

## Abstract

The prevalence of atrial fibrillation (AF), which is one of the common arrhythmias in clinics, is increasing sharply and has affected millions of patients, which is expected to triple by 2050. The purpose of the study was to explore the regulatory relationship between Src-homology domain 2 containing protein tyrosine phosphatase-1 (SHP-1) and proto-oncogene tyrosine-protein kinase Src (c-Src) and the regulation of Connexins 43 (Cx43), and its effect on AF was also studied. Mouse atrial myocyte line (HL-1 cell line) was used as the research object. After overexpression of SHP-1, the expressions of p-c-Src, Cx43, and SHP-1 were detected by Western blot and cellular immunofluorescence, respectively. The location and interaction of SHP-1 and c-Src in the cells were detected by immunofluorescence co-localization and co-immunoprecipitation (Co-IP). The regulation of c-Src and Cx43 was detected by DNA pull down, chromatin co-immunoprecipitation (CHIP), and dual-luciferase reporter system. The results revealed that overexpression of SHP-1 could inhibit the phosphorylation and activation of c-Src and increase the expression of Cx43. Moreover, there was a direct binding between SHP-1 and c-Src, and c-Src could bind to the promoter region of Cx43 and inhibit the transcription of Cx43. In conclusion, SHP-1 could bind to c-Src and inhibit the activity of c-Src, thus enhancing the transcriptional activation of Cx43 and improving the function of gap junction.

## Highlights

- SHP-1 inhibits the phosphorylation and activation of c-Src.
- SHP-1 increases the expression of Cx43.
- C-Src binds to the promoter region of Cx43 and inhibit the transcription of Cx43.

## 1 Introduction

Atrial fibrillation (AF) is one of the common arrhythmias in clinics. With the increase in age, the prevalence of AF increases sharply, from about 1% of the general population to about 10% of people over 80 years old [1,2]. At present, millions of patients are affected by AF that is expected to triple by 2050 [3]. AF can easily lead to thrombosis and increased ventricular rate, which is the main cause of embolic stroke. It is estimated that about 15% of strokes are associated with atrial fibrillation [4]. Atrial fibrillation affects the quality of life in patients and brings a huge economic burden to the whole society [4].

RETRACTED

Gap junction communication is essential in the electrical conduction between cardiac tissues, mediating the transmission of action potential between cells and coordinating myocardial electrical activity. Gap junction protein (connexins) is the main protein that constitutes connectors and gap junctions [5]. Connexins 43 (Cx43) is one of the main gap junction proteins in atrial myocytes. It plays an important role in the occurrence and maintenance of arrhythmias [6]. Src-homology domain 2 containing protein tyrosine phosphatase-1 (SHP-1) is a non-receptor protein tyrosine phosphatase, which is mainly expressed in hematopoietic cells and epithelial cells. As a negative regulatory factor, SHP-1 participates in a variety of signal pathways in eukaryotic cells, which is responsible for controlling the reduction and termination of signal cascade reactions [7]. The proto-oncogene tyrosine-protein kinase Src (c-Src) is an important member of the Src kinase family. It is a non-receptor tyrosine kinase and can be activated by multiple signal transduction pathways and then activate the corresponding signal pathways [8]. Studies have shown that c-Src protein plays an important role in normal cell mitosis, tumorigenesis, and metastasis [9]. The excess activation of angiotensin can mediate the process of cardiac remodeling that can be influenced by connexin and thus makes the connexin crucial in the occurrence and development of atrial fibrillation [10]. The excess activation of renin–angiotensin system directly leads to the activation of c-Src, and then c-Src mediates the decrease of Cx43 protein expression [11].

In our previous study, we found that angiotensin-(1-7) [Ang- (1–7)] could promote the expression of SHP-1, which is instrumental in regulating c-Src and antagonize the effect of Cx43 remodeling induced by angiotensin [12]. We speculated that SHP-1 might affect the expression of Cx43 through the regulation of c-Src, thereby participating in the regulation of atrial fibrillation. In order to further clarify the regulatory mechanism of SHP-1 and c-Src on Cx43 and their effects on atrial connexin remodeling, we explored whether the interaction between SHP-1 and c-Src is the central link of Cx43 expression and function in mouse atrial myocyte line HL-1 cells.

RETRACTED

## 2 Materials and methods

### 2.1 Cell culture and cell transfection

HL-1 cells were purchased from ATCC (American Type Culture Collection, USA). In order to maintain atrial contractility and stable passage of HL-1 cells, the cells were inoculated in a culture flask containing gelatin/fibronectin and added with Claycomb medium and 10% fetal bovine serum, 100 U/mL penicillin/streptomycin, 0.1 mmol/L norepinephrine, and 2 mmol/L L-glutamine. The culture was carried out in a 37°C incubator containing 5% CO_2_, and the liquid was changed every 24–48 h. SHP-1 overexpression lentivirus was constructed and packaged by Chongqing BioMedicine Biotechnology Co., Ltd and the empty vector was used for control. When the cells were infected, the virus concentration was 1 × 10^7^. After 48 h of virus infection, cell samples were collected for detection [13].

### 2.2 Western blot detection

HL-1 cells were intervened by different intervention groups, then the lysate was added, and the supernatant was obtained by 30 min, 13,800× g centrifugation for 15 min. The protein concentration was determined by the bicinchoninic acid (BCA) method, diluted with 5× sample buffer, and boiled for 5 min at 100°C. Prepare 10% SDS–polyacrylamide gel to separate protein and then transfer protein to polyvinylidene fluoride (PVDF) membrane. Primary antibodies used were as follows: anti-Cx43 (1:8000), anti-p-c-Src (1:1000), anti-SHP-1 (1:1000, Proteintech), anti-GAPDH (1:1000, Beyotime) as the internal control. The secondary antibodies of the corresponding species were incubated at room temperature for 1 h after washing the membrane with Tris-buffered saline with 0.1% Tween 20 (TBST) for 3 times and 10 min, each time [14]. TBST membrane was washed 3 times, 10 min, each time, and enhanced chemiluminescence reaction solution was added. The quantitative analysis of the bands was carried out by Image Lab Software.

### 2.3 qPCR detection

The reverse transcription reaction was carried out according to TAKARA kit. The reaction system was RNA, 2.2 μg; OligodT, 2 μL; dNTP, 4 μL; 5× buffer, 4 μ L; Reverse Transcriptase, 1 μL; RNAase inhibitor, 0.5 μL; RNAase free ddH_2_O, up to 20 μL. The reaction conditions are 25°C, 5 min, 50°C, 15 min, 85°C, 5 min, 4°C, 10 min.

The qPCR experiment was carried out according to the Optimo qPCR kit. The reaction system included forward primer, 0.4 μL, reverse primer, 0.4 μL, SYBRGreen, 10 μL, H_2_O 5.2 μL. The reaction conditions are 50°C, 2 min, 95°C, 10 min, 95°C, 30 s, 60°C, 30 min, 40 min. The primer of SHP-1 was SHP-1-F, 5’-GGTCACCCACATCAAGGTCAT-3’; SHP-1-R, 5’-TGTCGAAGGTCTCCAAACCAC-3’. The Cx43 primer was Cx43-F, 5’-CCCCACTCTCACCTATGTCTCC-3’; and Cx43-R, 5’-ACTTTTGCCGCCTAGCTATCCC-3’ [15].

RETRACTED

### 2.4 Cell immunofluorescence detection

HL-1 cells were fixed with 4% paraformaldehyde for 15 min, rinsed with PBS 3 times, 5 min for each time, and sealed with immunofluorescent blocking solution (Beyotime, QUICK BLOCK) for 15 min [16]. The primary antibody used was as follows: anti-Cx43 (1:500, Abcam), anti-p-c-Src (1:500, CST), and anti-SHP-1 (1:500, Proteintech). Then, cells were incubated with the fluorescent secondary antibodies (1:200, Dylight-594 goat anti-rabbit IgG and goat anti-human IgG) at darkroom temperature for 1 h. The nuclei were restained with DAPI for 15 min. The cells were washed with PBS 3 times, 5 min each. The tablets were sealed with an anti-fluorescence quenching agent, observed, and photographed under a fluorescence microscope.

### 2.5 Co-IP test

The cells were lysed with RIPA lysis buffer. 50% Protein A/G agarose working solution was added to the sample in the proportion of 100 μL per 1 mL. Shake the mixture in the horizontal shaker for 10 min at 4°C. 14,000 g centrifugation for 15 min at 4°C. The supernatant was transferred to a new centrifuge tube to remove protein A/G-agarose microspheres. The concentration of total protein was determined by BCA methods. SHP-1 or c-Src primary antibody was added, and at the same time, the Rabbit IgG polyclonal antibody (30,000-0-AP; Proteintech) was added as the control. The mixture was shaken slowly in a shaker, overnight at 4°C. The supernatant was collected for Western blot analysis [17].

### 2.6 DNA pull down

The Cx43 promoter region labeled with biotin was synthesized by Tsingke Biotechnology Co., Ltd. According to the DNA pull down kit (GZSCBIO, China) instructions, 5 μg biotin-labeled DNA and 500 μg total cellular protein were pre-mixed and placed on ice. 100 μL Streptavidin-agarose G magnetic beads was added to the mixture, incubated at 4°C for 1 h, centrifuged at 5000 g for 30 s; the supernatant was removed; the precipitation was collected; and 30 μL protein was added to the sample buffer [18].

### 2.7 Chromatin immunoprecipitation test (CHIP)

The chromatin immunoprecipitation was performed using Pierce Agarose ChIP Kit (Thermo Fisher Scientific). The total cell protein was cross-linked with 1% formaldehyde for 15 minutes before homogenizing. The DNA was cut to 200-1000 bp by ultrasonic crushing apparatus. c-Src antibody was added and incubated at 4°C overnight. The cross-linking was reversed at 65°C for 8–10 h to obtain the DNA [19].

### 2.8 Double luciferase reporting system detection

The PGL3-CX43-promoter luc carrier and pcDNA3.1-c-SRC carrier were synthesized and constructed by Chongqing Biomedicine Biotechnology Co., LTD. Cell transfection was carried out according to routine operation, and plasmids of each group were transfected into cells using Lipo2000. PGL3-Basic plasmid and pRL-TK control vector were co-transfected into cells as control. Twenty-four hours later, firefly luciferase and renilla luciferase activities were detected according to the dual-luciferase reporting system assay kit (Promega, USA) [20].

RETRACTED

### 2.9 Statistical treatment

SPSS 20.0 software was used for statistical analysis of the experimental data. The measurement data were expressed as mean ± standard error (X ± s). T-test was used for comparison between two groups. P < 0.01 was considered as very significant difference.

## 3 Results

The purpose of this study was to explore the regulatory relationship between SHP-1 and c-Src and to study its regulatory effect on Cx43 and the effect of atrial fibrillation. The hypothesis is that SHP-1 might affect the expression of Cx43 through the regulation of c-Src, thereby participating in the regulation of atrial fibrillation. After over-expression of SHP-1, the expressions of p-c-Src, Cx43, and SHP-1 in HL-1 cells were detected by Western blot and immunofluorescence. The regulatory effects of c-Src and Cx43 were detected by DNA pull down, chromatin immunoprecipitation, and dual-luciferase reporter system.

### 3.1 Overexpression of SHP-1 inhibits the activation of c-Src and increases the expression of Cx43

After the overexpression of SHP-1 in HL-1 cells cultured in vitro, qPCR and Western blot were performed to detect the expression of genes. As shown in Figure 1(a), the relative gene expression of SHP-1 and Cx43 in OE-SHP-1 was elevated remarkably compared with NC (P < 0.01). It showed that in contrast to NC, the protein expression levels of SHP-1 and Cx43 were significantly increased in OE-SHP-1 (P < 0.01), while the protein expression of p-c-Src was significantly decreased (P < 0.01, Figure 1(b)). The expression levels of SHP-1, Cx43 and p-c-Scr were also detected by cellular immunofluorescence. The results showed that the expression levels of SHP-1 and Cx43 were increased after overexpression of SHP-1, while the expression levels of p-c-Scr were significantly decreased after overexpression of SHP-1 (P < 0.01, Figure 2(a-2b)). This result was consistent with our previous results of adding Ang-(1-7) [12].

**Figure 1.** SHP-1, c-Src, p-c-Src, and Cx43 expression after overexpression of SHP-1 was detected by qPCR and western blot. (a) qPCR was used to detect the gene expression of SHP-1 and Cx43 in HL-1 cells. (b) The expression of SHP-1, c-Src, p-c-Src, and Cx43 in HL-1 cells was detected by WB, and semi-quantitative analysis based on gray value was performed. OE-SHP-1, HL-1 cells transfected with SHP-1 overexpression lentivirus. NC, HL-1 cells transfected with lentivirus vector. ##, p < 0.01.

RETRACTED

**Figure 2.** The protein expression after overexpression of SHP-1 was detected by immunofluorescence. (a) The microscopy images of SHP-1, p-c-Src, and Cx43 stained in HL-1 cells were photographed under a fluorescence microscope. (b) The average fluorescence intensity was calculated. OE-SHP-1, HL-1 cells transfected with SHP-1 overexpression lentivirus. NC, HL-1 cells transfected with lentivirus vector. ##, p < 0.01. Scale bar: 50 μm.

### 3.2 Direct combination of SHP-1 and c-Src

In order to clarify the regulatory mechanism of SHP-1 on c-Src, it was found that c-Src and SHP-1 were co-located in cells by immunofluorescence (Figure 3(a)). Furthermore, by Co-IP test, it was found that c-Src could be detected in the protein complex pulled down by SHP-1 antibody (Figure 3(b)). And SHP-1 protein could also be detected in the protein complex pulled by c-Src antibody (Figure 3(c)). This showed that c-Src and SHP-1 could bind directly in the cell. After overexpression of SHP-1, the phosphorylation level of c-Src decreased and the expression of its downstream protein Cx43 increased (Figure 1(b)), indicating that the binding of SHP-1 to c-Src could inhibit the phosphorylation of c-Src and its activity, thus enhancing the transcriptional activation of downstream genes.

**Figure 3.** SHP-1 is directly combined with c-Src. (a) The immunofluorescence co-localization of SHP-1 and c-Src protein in HL-1 cells. Scale bar: 50 μm. (b) Co-IP test was performed with SHP-1 antibody and cell extract co-precipitated IgG polyclonal antibody was used as control, and the cell extract was set as an input. (c) Co-IP test was performed with c-Src antibody and cell extract co-precipitated IgG polyclonal antibody was used as control, and the cell extract was set as an input.

### 3.3 c-Src binds to the promoter region of Cx43 to inhibit its transcription

Next, in order to further explore the molecular regulatory mechanism of SHP-1, the upstream 2000 bp sequence of the transcriptional initiation site of Cx43 was obtained from the UCSC database (genome-asia.ucsc.edu), and the transcription factors that might bind to the Cx43 promoter region were predicted in the HumanTFDB database (bioinfo.life.hust.edu.cn). The results showed that the Cx43 promoter region consisted of three c-Src binding sites, indicating that c-Src might bind to the Cx43 promoter region to regulate its transcription. In order to further clarify the transcriptional regulation of c-Src on Cx43, we detected it by dual-luciferase reporter system and found that c-Src inhibited the transcriptional activation of Cx43 promoter (Figure 4(a)). In order to prove the binding effect of c-Src and Cx43 promoter more accurately, we verified it by DNA pull down and CHIP tests. Consistent with our prediction, the c-Src protein was detected in the Cx43 promoter region by DNA pull down test, and the DNA fragment pulled by CHIP was amplified by multiple pairs of primers, and the positive sequence was successfully cloned by two pairs of primers (Figure 4(b-c)). These results suggested that c-Src could bind to the promoter region of Cx43 and inhibit its transcriptional process.

RETRACTED

**Figure 4.** C-Src binds to the promoter region of Cx43 to inhibit its transcription. (a) The double-luciferase reporter system was used to detect the regulation of c-Src on Cx43 promoter. (b) The binding of c-Src and Cx43 DNA was detected by DNA pull down. (c) The binding effect of c-Src and Cx43 DNA was detected by chip. M, DL2000 marker; 1–5, negative primers; 6–7, positive primers.

## 4 Discussion

Cx43 is an important junction protein of adjacent cardiomyocytes. Connexin remodeling is an important part of atrial myoelectric remodeling and an important cause of atrial conduction delay and anisotropy [21,22]. Changes in the number and distribution of Cx43 are the molecular anatomical basis of myocardial remodeling and arrhythmias. The heart conduction velocity of mice without Cx43 is slow, which can easily lead to arrhythmia death [23,24]. In the process of myocardial ischemia or myocardial injury and fibrosis, the expression of Cx43 will decrease, resulting in electrophysiological remodeling of cardiomyocytes at the molecular level, leading to arrhythmia [25,26]. Moreover, the study has revealed that Cx43 reduces susceptibility to sympathetic atrial fibrillation [27]. In this study, it was found that after overexpression of SHP-1, the expression of Cx43 was significantly increased, indicating that SHP-1 can reduce myocardial fibrosis and effectively protect myocardial function. This is consistent with the previous research results in this project, which antagonized the activation of c-Src mediated by Angiotensin II (AngII) by increasing the expression of SHP-1 by adding Ang- (1–7), and then antagonized the atrial connexin remodeling induced by AngII, and finally showed antiarrhythmic effect [12].

C-Src exists widely in cardiomyocytes and participates in AngII signal transduction. AngII directly leads to the activation of c-Src, which mediates the decrease of Cx43 protein expression induced by AngII [28]. In the early stage of this project, through the intervention of cells with the addition of AngII, it was found that it could inhibit the expression of Cx43. At this concentration, it did not affect the activity of cardiomyocytes, but the activity of c-Src increased significantly, while the degree of inhibition of Cx43 was the most obvious. Inhibition of c-Src can reverse this effect of AngII, improve the expression of Cx43 protein after myocardial infarction, and reduce the occurrence of ventricular arrhythmias [29]. In this study, it was proved that c-Src can bind to the promoter region of Cx43 to regulate its transcriptional activity. Through direct overexpression of SHP-1, it was found that the expression of p-c-Src protein decreased significantly, and the expression of its downstream protein Cx43 increased, indicating that the binding of SHP-1 to c-Src can inhibit the phosphorylation of c-Src and inhibit its activity, thus enhancing the transcriptional activation of downstream genes.

RETRACTED

SHP-1 regulates protein status by dephosphorylation, usually by inhibiting protein activity. Previous studies have suggested that the Ang-(1-7)/Mas axis may negatively regulate the activation of c-Src and its downstream signals induced by AngII by enhancing the SHP-1 activity of renal proximal convoluted tubule cells [30]. When the tyrosine phosphatase inhibitor was added to the previous study of this project, compared with AngII+Ang-(1-7) group, the expression of SHP-1 decreased significantly. On the contrary, the activity of c-Src increased, which finally showed that the expression of Cx43 decreased and the intercellular transmission function was impaired [31]. It is suggested that Ang-(1-7) antagonizes the inhibitory effect of AngII on Cx43 and recovers the expression of Cx43 by inhibiting the activity of c-Src by SHP-1. Thus, the increased expression of SHP-1 can improve the efficiency of intercellular transmission. Ang-(1-7) antagonizes the activation of c-Src mediated by AngII by increasing the expression of SHP-1, and then antagonizes the connexin remodeling of atrial muscle induced by AngII, and finally shows antiarrhythmic effect [30–32]. Studies have confirmed that renin–angiotensin system (RAS) inhibitors can reduce the load of atrial fibrillation to some extent, delay the progression of the disease to persistent atrial fibrillation, regulate the expression and functional status of connexin, and inhibit the abnormal distribution of connexin in a pathological state [33,34]. ACE2/Ang-(1-7)/Mas, as the most important endogenous regulatory axis of RAS, plays an important role in the negative regulation of AngII-mediated myocardial remodeling [35]. In the previous study of rat cardiac fibroblasts, it was found that Ang- (1–7) could limit the activation of ERK induced by AngII by activating SHP-1, further inhibiting the production of TGF-β and collagen, and show the effect of anti-myocardial fibrosis [12]. This study also confirmed that overexpression of SHP-1 could reduce the level of phosphorylation and activation of c-Src and increase the expression of Cx43. There was a direct binding between SHP-1 and c-Src. c-Src could bind to the promoter region of Cx43 and inhibit the transcription of Cx43. This study further revealed the regulatory relationship between SHP-1/c-Src/Cx43 and the molecular regulatory mechanism, which provided a basis for further understanding of connexin and the treatment of atrial fibrillation. Since the experiments in this study were performed on cells cultured in vitro and were not further verified in animal models, this study still has some limitations. In future research, we will further study this mechanism at the animal level, and further verify the molecular regulation mechanism using gene editing methods to knock out genes.

RETRACTED

## 5 Conclusion

There is a direct binding between SHP-1 and c-Src. C-Src can bind to the promoter region of Cx43 and inhibit the transcription of Cx43. SHP-1 inhibits the activity of c-Src, increases the expression of Cx43, and improves the function of gap junction.
